# Path Deconstruction of Agricultural Environmental Sustainable Development Policy in the Process of International Agricultural Trade Liberalization

**DOI:** 10.1155/2022/3101244

**Published:** 2022-09-28

**Authors:** Xiaozhong Li, Feng Huang

**Affiliations:** ^1^Academy of Green Food Science of Heilongjiang, Northeast Agricultural University, Harbin 150030, Heilongjiang, China; ^2^College of Economics and Management, Northeast Agricultural University, Harbin 150030, Heilongjiang, China

## Abstract

Agriculture is particularly essential in the equilibrium between man and nature because of its intimate contact with nature. So the cornerstone for the sustainable development of the human economy and society is the sustainable development of agriculture. When it comes to global trade, agricultural trade has always been in a very special position. The basic situation of agriculture involves food safety, environmental protection, Chinese politics, and many other issues. In order to overcome the problems of overlapping, repetitive, and too many indicators in the evaluation method of agricultural environmental sustainable development and unfavorable for practical operation, this paper proposes an ecological footprint model based on emergy. The model can effectively evaluate the ability of sustainable development of agricultural environment and solve the problem that traditional evaluation methods cannot comprehensively evaluate. This makes agricultural development sustainable and is conducive to the liberalization of international agricultural trade. The experimental results of this paper show that from 2014 to 2018, the degree of damage to the agricultural environment has increased from 21% to 45%, which has led to a decline in the quality of agricultural products, and the output and sales are not as good as before. It can be seen that only by ensuring the sustainable development of the agricultural environment can we ensure the smooth progress of the international agricultural trade liberalization and make China's economy flourish.

## 1. Introduction

Carrying out the protection of agricultural environment has an inestimable value for the development of agriculture, and it is beneficial to the continuous development of China's economy. The agricultural sector is an important production sector in China, providing people with a variety of means of life and production, and has become the basis for the development of the national economy. Agricultural production refers to the use of natural resources such as land for production activities. The soil, water, atmosphere, etc., in the natural environment are important resources for agricultural production, as well as major environmental factors. Due to the objective reasons that the Chinese people have more land and less land, in order to solve the problem of people's food and clothing, and face the pressure of people's growing material demand, people's activities are all oriented to the pursuit of grain production. Scholars began to explore whether the agroecological environment was affected. As an open system, the production mode of agriculture itself and some internal and external factors of agriculture have certain influence on the agroecological environment. After decades of practice, people will find that the environmental capacity is limited. In order to realize the sustainable development of agriculture, it is very important to ensure the sustainable development of the agricultural ecological environment.

With the close international exchanges, the improvement of China's agricultural internationalization and trade liberalization, and the changes in the market supply and demand structure of agricultural products, China has further deepened the foreign trade policy of agricultural products while implementing the strategic adjustment of agricultural products. The EU is China's first trading partner and has also gradually become China's major agricultural trade partner. China is a developing nation with quick economic expansion. China's economy has been more internationalized and significant in the global economy since the adoption of the reform and opening up program. Trade volume and impact on the global economy have risen steadily over time. Agricultural commerce has also increased in importance relative to other sectors of the Chinese economy. This paper's originality is its use of the emergy ecological footprint model to assess agricultural environment sustainability, identify issues with agricultural environment sustainability, and take proactive measures to address such issues. This makes it possible for agriculture to grow sustainably, guaranteeing the position of agricultural goods in the liberalization of global trade.

## 2. Related Work

Sustainable agroenvironmental development means that it is technically appropriate, economically feasible, and widely accepted by society, without deteriorating the environment and maintaining the development of land, water, and plant resources. The possible effects of agriculture trade liberalization on various nations were examined by Nuetah and Xin. To calculate the probable effect of agricultural trade liberalization on global agricultural market prices, they employed simulation models for agricultural trade and policy [1]. According to Sunge and Ngepah's research, China is now a net importer of agricultural products despite the growing liberalization of agricultural commerce. While neglecting the connection between efficiency, empirical research have concentrated on the relationship between trade liberalization and productivity development. They provided evidence that agricultural trade statistically increases technological efficiency through technology transfer [2]. Baer-Nawrocka et al. found that every reform of the Common Agricultural Policy (CAP) has some impact, not only on agricultural products but on society as a whole. They proposed a new methodology to determine the potential impact of EU agricultural policy reforms, which is combined with game theory [3]. Mensah et al. found that China has about 22% of the world's population and less than 10% of the arable land and faces many challenges in the agricultural sector. They discussed the main challenges facing China's agricultural sector and its future prospects. Urbanization, industrialization, environmental pollution, and trade liberalization are identified as the main problems facing China's agricultural sector [4]. According to Karunakaran and Sadiq, liberalization and modernization represent a serious danger to agriculture, which is the primary source of income for farmers. Organic farming is environmentally benign, supports sustainable development, maintains soil fertility, and gives farmers long-term crop income. By giving better pricing and enhancing the lives of their communities, free trade emerged as a movement to help disadvantaged organic farmers [5]. The importance of agriculture to China's economy has been discussed by academics. China is a sizable agricultural nation, and agriculture and economic development are inextricably linked. Additionally, the liberalization of commerce has a significant impact on agriculture, so it is very necessary to develop sustainable agriculture in order for China to maintain a pivotal position in the world. But the scholars did not mention how to make the agricultural environment sustainable.

In recent years, the free trade of international agricultural products is developing faster and faster, which also brings some problems to the agricultural environment. According to Yang and Hu, the evaluation of regional ecological construction is based on capital stock and capital flow use, which helps to encourage the coordinated growth of the economy and natural capital utilization and raise the effectiveness of that utilization. They applied the partial least squares method to determine the driving forces behind changes in the region's ecological footprint through the examination of per capita ecological footprint and per capita ecological carrying capacity [6]. Liu et al. believed that global warming is a very serious environmental problem. People have the responsibility to build a low-carbon agricultural environment, and they proposed a comprehensive model of ecological footprint. This indicates that the agroenvironment is classified as highly sustainable to promote agroenvironmental sustainability [7]. Ma et al. thought that the inconsistency between China's economy's rapid growth and its agricultural environment, which is not favorable to the sustainable development of agriculture, has become more pronounced. A common metric of sustainable growth is the ecological footprint. They made the emergy ecological footprint model his method of choice in an effort to address the sustainable development of the agricultural environment [8]. Using a recently created ecological footprint model, Aydin et al. investigated the nonlinear impacts of economic expansion on the ecological footprint as an indicator of environmental deterioration. According to empirical findings, environmental pressure on agriculture will rise as the economy develops [9]. Scholars have found that in the development of agriculture, the agricultural environment is facing important challenges. With the development of economy, the agricultural environment has also been destroyed. If people want sustainable development of agriculture, people should solve the problem of sustainable development of agricultural environment. Scholars use the ecological footprint model to evaluate the sustainable development of the agricultural environment and improve the unfavorable indicators. But scholars have no concrete measures to address this problem.

## 3. Based on the Ecological Footprint Model and Sustainable Development of Agricultural Environment

### 3.1. Relationship between Agricultural Environment and Sustainable Agricultural Development

The development of agriculture has further promoted the improvement of the world industry, the world economy, and the living standards of the world people. Agricultural productivity has increased rapidly due to the substantial increase in energy input, but it has also suffered from a series of serious ecological and environmental impacts [10]. This operation results in compaction of the soil and reduction of soil organic matter. On the one hand, the industry helps to realize agricultural mechanization and modernization; on the other hand, it causes pollution of water, atmosphere, and soil, which brings immeasurable losses to the agricultural ecological environment [11]. The sustainable development of agriculture is shown in Figure 1.

As shown in Figure 1, the sustainable development of agriculture requires a good ecological environment, which is not only a social and economic reproduction process but also a natural reproduction process of the production, development, and reproduction of animals and plants themselves. Sustainable agriculture is an agriculture that manages, protects and sustainably utilizes natural resources, adjusts farming systems and techniques, and continuously meets the needs of contemporary human beings for the quantity and quality of agricultural products without harming the interests of future generations. The agroecological environment and animals and plants are interdependent and affect each other and maintain a certain dynamic balance [12].

Agricultural natural reproduction has the characteristics of long cycle and dependence on seasonal, regional, and natural environment factors. Due to changes in environmental factors, it is easy to affect the quality of products. Therefore, agriculture is a weak industry, and its production cycle requires not only the support of external policies and equipment investment but also a good natural ecological environment for crops to grow. Agriculture is the economic lifeline of a country, and protecting the agricultural ecological environment is conducive to maintaining the sustainable development of agriculture and is conducive to farmers' food and clothing security. The agricultural environment is shown in Figure 2.

As shown in Figure 2, the sustainable development of agricultural environment is an extension of a globally recognized sustainable development strategy in the field of rural economic development. At present, the whole world is advocating the concept of sustainable development under the banner of sustainable development. The sustainable development of agriculture will also become the eternal theme of the world. Sustainable agricultural development is an agriculture that can maintain and rationally utilize land, water, and animal and plant resources without causing environmental degradation, while being technically feasible, economically viable, and widely accepted by society.

### 3.2. Evaluation Method of Agricultural Sustainability Index (ASDI)

Numerous research have demonstrated the existence of the phenomena of diminishing returns in the input of agroecosystems and the S-shaped relationship between the ecosystem's input and output. This means that the marginal productivity of the system is positively connected with input up to a certain level and starts to fall after that point [13]. Marginal productivity refers to the increase in output or revenue by adding the last unit of the factor of production, other things being equal. The environment supporting agriculture has the highest ecological carrying capacity. An excessive amount of input will result in a decrease in output, an inability to raise output, and environmental contamination. This study clarifies the input efficiency of agricultural production and assesses the state of sustainable development through the analysis of agricultural energy input and output.

The level of the farming ecosystem's energy input and output in an S-curve scenario can be used to assess the ecosystem's sustainability. Energy input and emissions are at an accelerated stage of declining marginal benefits when the input surpasses the carrying capacity of the largest ecosystem in the area. As a result, the Kuznets curve and the agricultural sustainable development index are similar [14]. The Kuznets curve is a hypothetical curve that depicts the relationship between economic inequality and per capita income in the process of economic development (assumed to be time-dependent).  Figure 3 displays the figure for the agricultural sustainable development index.

As shown in Figure 3: The S-curve is used in this study to determine the inflection point P of production and investment profits and to split the range of marginal revenue growth and decline. And use the parabolic first derivative as the critical point of energy investment, that is, to reach the maximum support force of the regional PK, to determine the investment required to increase the interval of negative ecological impact [15]. Internet energy investment is to help residents invest and trade in energy through the high-speed convergence of Internet information.

The specific methods include finding the corresponding means of production:

(1) $$\begin{array}{c} b=\frac{K}{1+e^{\left(ax+b\right)}}. \end{array}$$

The inflection point value P will appear if the limit productivity is equal to the average productivity, which is the case when EEI = 1, and the associated PA may be determined using the following formula:

(2) $$\begin{array}{c} AEP=\frac{\left(b-b^{0}\right)}{a},\\ MEP=\frac{db}{da}=-k\times \frac{a\times e^{\left(ax+b\right)}}{{\left(1+e^{\left(ax+b\right)}\right)}^{2}},\\ EEI=\frac{MEP}{AEP}. \end{array}$$

The sustainable development of agriculture is different from the sustainable development of other fields such as industry, and its index system should include its specific index. The Agricultural Sustainability Index (ASDI) is divided into three intervals, and the range of values is set between -1 and 1, such as follows:

(3) $$\begin{array}{c} ADSI=\left\{\begin{array}{c} \frac{A}{PA},\left(0,1\right]\\ \frac{E-A}{E-PA},\left(1,0\right]\\ \frac{E-A}{A},\left(0,-1\right]. \end{array}\right. \end{array}$$

### 3.3. Ecological Footprint Model

Ecological footprint analysis is a biological method to measure the degree of sustainable development. Ecological footprint is the biologically productive territorial space that can continuously provide resources or consume waste. In the resource environment system, whether it is human survival and development, or the accommodation of resource exploitation and waste, it needs to occupy a certain environmental space. And this kind of space with resource production function and waste storage function is ecological productive land [16], as shown in Figure 4.

As shown in Figure 4, the productive land that can provide agricultural products, livestock products, timber, fishery products, and urban residential areas and roads is called the ecological footprint of biological resources. It is composed of the total ecological demand of cultivated land, grassland, woodland, water area, and construction land [17, 18].

The model of the ecological footprint analysis method is as follows:

(4) $$\begin{array}{c} EF=Nef=N\overset{n}{\underset{i=1}{\sum }}\left(\frac{rici}{pi}\right). \end{array}$$

In the formula, *i* represents the category of consumer goods, and EF represents the sum of the ecological footprint. In the calculation of ecological environment capacity, due to the difference of resource stock and ecological productivity in each region, the adjustment must be multiplied by the corresponding balance coefficient. The proposal of ecological carrying capacity is a great progress for the study of carrying capacity theory. Compared with single-factor carrying capacity, ecological carrying capacity pays more attention to the integration, sustainability, and coordination of ecosystems. The calculation formula of ecological carrying capacity is as follows:

(5) $$\begin{array}{c} EC=NeC=N\overset{6}{\underset{i=1}{\sum }}\left(aj\times rj\times yj\right). \end{array}$$

*yj* is the yield factor of different types of ecologically productive land.

The ecological footprint model is easy to understand, the calculation method is simple, and the calculation results are quantified, so that people can intuitively perceive the degree of impact on the environment [19]. At the same time, the ease of comparison with the limited supply of Earth's space makes the measure of sustainable development truly regionally comparable.

Although the ecological footprint model has many advantages, it still has many shortcomings. It is mainly manifested in that the research method is only based on ecology and does not fully reflect the actual resource occupation of the ecological environment by human beings [20].

### 3.4. Ecological Footprint Model Based on Emergy Deconstruction

The proposal of the concept of sustainable development has aroused great repercussions from the international community, prompting scholars to conduct in-depth research on its evaluation system and analysis methods. Using a certain index system to scientifically evaluate the status and effect of regional sustainable development and provide reasonable theoretical guidance and policy recommendations for sustainable development in different regions has become a hot topic of current research.

Emergy analysis method is mainly used in the evaluation of ecological benefits, used in the study of ecosystems and human social and economic systems, and quantitatively analyzes the real value of resources, environment, and economic activities and the relationship between them. And it improves the approaches used in research on the evaluation of sustainable development.

The status of sustainable development can be reflected by the results obtained by comparing the ecological footprint and ecological carrying capacity. The calculation formulas are as follows:

(6) $$\begin{array}{c} ER=EC-EF,\\ ED=\frac{EC}{EF}. \end{array}$$

In the formula, *ER* represents ecological surplus, and *EC* represents ecological deficit. The formula for calculating the per capita ecological footprint is

(7) $$\begin{array}{c} E_{f}=\overset{n}{\underset{i=1}{\sum }}a_{i}=\overset{n}{\underset{i=1}{\sum }}\frac{c_{i}}{p_{2}}. \end{array}$$

Among them, *E*_*f*_ is the per capita ecological footprint, and *a*_*i*_ is the per capita ecological footprint of the *i*th resource.

For renewable resources, the sustainable utilization of resources is mainly achieved by reasonably regulating the utilization rate of resources. The sustainable utilization of renewable resources is mainly restricted by the law of natural growth. When calculating the ecological environment carrying capacity, only the use of renewable resources can make the ecological environment carrying capacity truly sustainable, as shown in the following:

(8) $$\begin{array}{c} E_{c}=\frac{e}{p_{1}}. \end{array}$$

Among them, *E*_*c*_ is the per capita ecological carrying capacity, *e* is the per capita solar energy value of renewable resources, and *p*_1_ is the global average emergy density.

Add a person's ecological footprint to each consumer item and compare it with each person's ecological capacity. Using this, we measure the ecological profit and loss of the region:

(9) $$\begin{array}{c} E_{p}=E_{c}-E_{f}. \end{array}$$

If *E*_*p*_≻0, it means that there is an ecological surplus, and the regional ecosystem is in a sustainable state.

Ecological profit and loss refers to the difference between ecological carrying capacity and ecological footprint, and this index indicates the ecological status of a certain area. The calculation of ecological profit and loss can directly reflect the carrying status of the development of the research area, but the degree of utilization of natural resources in the area needs to be measured by the sustainable development index. Its calculation method is as follows:

(10) $$\begin{array}{c} SEI=\frac{E_{c}}{\left(E_{c}+E_{f}\right)}. \end{array}$$

The ecological footprint diversity index is used to represent the ecological footprint balance of different consumer goods in the survey area. The calculation formula is

(11) $$\begin{array}{c} H=-\sum \left(P_{i}\times {InP}_{i}\right). \end{array}$$

Among them, *P*_*i*_ and *InP*_*i*_ represent the proportion and distribution of the ecological footprint of the *i*th consumption item in the total.

This paper mainly considers three kinds of renewable energy sources: solar radiation energy, rain chemical energy, and surface soil energy. Its calculation formula is

(12) $$\begin{array}{c} EC=\frac{E}{N\times D}\times B. \end{array}$$

In the formula, *EC* is the ecological environment capacity of per capita cultivated land, and *E* is the energy value of renewable resources on the surface of cultivated land in the survey area. The yield coefficients of various crops are summed using the weighted method to obtain the corrected field yield coefficients. The weights are different weights taken in the adjustment calculation due to the difference in the precision of the measured values. The higher the precision, the greater the weight. “Weighted” means “multiplied by the weight”, that is, “multiplied by the coefficient,” as shown in the following:

(13) $$\begin{array}{c} B=\sum \left(\frac{a_{i}}{G_{i}}\times p_{i}\right). \end{array}$$

*a*_*i*_ is the city (or county) average arable land yield of the *i*th crop.

## 4. Investigation and Deconstruction Based on Sustainable Development of Agricultural Environment

### 4.1. Investigation on the Development Trend of International Agricultural Trade Liberalization

After the implementation of the reform and opening policy, with the change of China's trade policy, the role and status of agricultural trade have also undergone fundamental changes. For a long time, China's agricultural trade has basically been in a surplus state. But by the late 1990s, the situation began to reverse, with surpluses and deficits alternating. The main purpose of agricultural trade is no longer to earn foreign exchange, but to gradually evolve to satisfy people's different consumption preferences to improve their quality of life, and at the same time, it is also conducive to the further improvement of farmers' income.

China's entry into the World Trade Organization is a new milestone for China's agricultural trade. With the changes in the market supply and demand of agricultural products, agricultural products gradually turn from shortage to surplus, which forces people to seek a channel to solve the surplus of agricultural products. Generally speaking, besides agricultural producers adjusting their own production structure and stimulating Chinese consumption to boost demand, seeking more trading partners to increase overseas exports is also an important way to solve the surplus of agricultural products. The import value of agricultural products is shown in Table 1.

As shown in Table 1, the growth rates of imports of cereals, vegetables, fruits, and livestock products in 2014 were 9.6%, 11.9%, 13.7%, and 16.2%, respectively. It can be seen that in 2014, China's agricultural products began to be initially imported. The growth rates of imports of cereals, vegetables, fruits, and livestock products in 2015 were 11.8%, 17.4%, 17.6%, and 18.5%, respectively. By 2018, the growth rates of imports of cereals, vegetables, fruits, and livestock products were 21.7%, 25.6%, 31.8%, and 23.3%, respectively. Compared with 2014, the growth rate has become much faster, which also shows that China's agricultural free trade has been developed.

The export value of agricultural products from 2014 to 2018 is shown in Table 2.

As shown in Table 2, in 2014, the growth rates of export value of cereals, vegetables, fruits, and livestock products were 5.7%, 8.7%, 11.9%, and 15.5%, respectively. It can be seen that in 2014, the development of China's agricultural product exports lagged behind the development of imports. By 2016, the export value of China's agricultural products began to catch up with the growth rate of the import value. By 2018, the growth rates of imports of cereals, vegetables, fruits, and livestock products were 33.2%, 35.5%, 33.0%, and 30.8%, respectively. Compared with the growth rate of imports, the growth rate increased by 11.5%, 9.9%, 1.2%, and 7.5%, respectively. At this time, it shows that China's agricultural products have been welcomed by the international community.

From the perspective of changes in agricultural output, due to the reduction of trade barriers, the role of comparative advantage in the adjustment of agricultural production structure is more obvious. Among all agricultural products, the increase rate and absolute amount of grain and fruit and vegetable production are the highest. Fruit and vegetable agricultural products have always been China's dominant agricultural products. And China's grain, especially rice, will increase its export demand due to the reduction of trade barriers, which will lead to the enhancement of its competitive advantage. This will promote the production of rice in China, which in turn will increase the total grain output, as shown in Figure 5.

As shown in Figure 5, the total income of farmers is increasing, but it is mainly concentrated in the fields of grains, fruits, vegetables, and meat. These agricultural products are also agricultural products with rapid export and output value growth. On the contrary, the income of cotton, oil crops, and vegetable oil workers has declined. This is because these agricultural products belong to the industries whose production is affected by the agricultural products of other countries, but because the impact is not large, the degree of income decline is not obvious. The employment situation of farmers from 2014 to 2018 is shown in Figure 6.

As shown in Figure 6, changes in farmers' income also bring corresponding changes in farmers' employment. The employment level of agricultural products with increased farmers' income also increased, and the employment level of farmers in the two sectors of fruits, vegetables, and meat increased the most. Due to China's sustained economic growth and a considerable scale of agricultural trade, the EU is optimistic about the international trade of agricultural products between the two sides. On the other hand, according to linked research, changes in the consumption pattern of agricultural products by EU citizens have occurred as a result of people's increased focus on their health, primarily seen in the rise in consumption of pork and poultry meat as well as the rising demand for agricultural goods like rice and edible fungus.

### 4.2. Investigation on Sustainable Development of Agricultural Environment in Province A

The agricultural production in province A mainly uses natural resources such as soil, water, etc., as well as a large amount of agricultural chemicals for production. The pursuit of pure grain yield is a simple linear development of “resources-production-products+waste.” This mode of production does not take into account the agroecological environment and does not pay enough attention to the environment.

The ecological environment of agriculture is the material basis of agricultural production, and it is also a major issue related to the development of contemporary agriculture, which is of strategic importance in the entire economic construction. As 70% of China's population lives in rural areas, it is very important to ensure and improve the quality of life of rural people. Its condition also determines the output, quality, and production potential of agricultural products and directly and indirectly affects the physical and mental health of human beings, which will inevitably affect the sustainable development of agriculture. Agriculture is an open system. Due to the pollution of agriculture itself, the pollution of industry, and the pollution of domestic waste, the agricultural ecological environment has been under triple pressure, and agricultural production has been affected. The national and provincial annual chemical fertilizer usage from 2014 to 2018 is shown in Table 3.

As shown in Table 3, in recent years, the increase in the application intensity of chemical fertilizers has begun to slow down, and the application rate of chemical fertilizers has reached a high level.

In addition to the excessive use of chemical fertilizers, the use of chemical fertilizers has had a certain impact on the agricultural ecological environment due to the unreasonable fertilization structure and the reasons for scientific fertilization. The effective utilization rate of chemical fertilizer is shown in Figure 7.

The harm and pollution trend of China's agroecological environment has not been substantially managed, as indicated in Figure 7, and certain places are continuously degrading. As a result, people must focus on preserving the sustainable growth of the agroecological environment that influences the quality of agricultural goods in order to compete with the market for high-quality agricultural products in China and overseas.

The change of China's agricultural free trade policy not only has an impact on the trade, production, and income of agricultural products industry sector itself but also has a significant impact on the environment. The agricultural environmental damage rate of province A in recent years is shown in Figure 8.

As shown in Figure 8, the impact of human activities on the environment has received increasing attention in countries around the world. Agriculture is an ecological and economic organism in which natural ecology and socioeconomics are interdependent, combined, changed, and interacted. Therefore, since the 1990s, the Chinese government has attached great importance to environmental protection and sustainable agricultural development and regarded it as an important goal of agricultural support policies.

### 4.3. Advocating the Concept of Sustainable Development of Agricultural Ecological Environment

From the strategic height of macrocontrol, develop relevant technical systems, policies, and legal support to comprehensively improve the rural ecological environment and promote agricultural development. In order to establish the view that environment is resource, environment is benefit, and environment is productivity, people realize that agriculture is not only the source of agricultural products but also the source of environmental services and the importance of agroecological environment. Farmers are the main body of agricultural production. Protecting the agricultural ecological environment and preventing agricultural pollution require the active participation of farmers. In order to make most farmers aware of the long-term benefits of the agricultural environment, it is necessary to strengthen publicity activities in the vast rural areas to improve people's environmental awareness and awareness of sustainable development.

#### 4.3.1. Change Production Methods and Develop Circular Economy

The current agricultural development model is a linear economic model, pursuing pure grain production, high-intensity development of the earth's materials and energy. This mode of agricultural development not only is not the best economic interests but also cannot achieve sustainable development from the perspective of environmental and ecological interests. Recently, the newly advocated development model is the closed-loop model of “resources-production-products + waste utilization-products,” which regards the reuse of agricultural wastes as the input of other agricultural industries. This model can achieve the win-win goals of the highest resource utilization rate, the lowest emission, and a virtuous circle of economy and ecology and basically realize the economic model of the transformation of China's agricultural model from a linear economic model to a circular economy.

#### 4.3.2. Adhere to the Dualism of Economic Development and Environmental Protection

It is essential to rationally use natural resources, reduce or avoid environmental pollution and ecological hazards, strengthen the prevention and management of environmental pollution, and enhance environmental quality in order to fully utilize the environment and natural resources during the process of economic development, then promote the sustainable growth of the social economy while realizing the sustainable development of the agricultural environment. Protecting the environment is a basic method to enable people and the environment to coordinate and develop sustainably, and its essence lies in ensuring the better development of productive forces. Agricultural environmental protection needs to cooperate with other countries and regions in the world, absorb the most advanced technology and the best production and living experience, and promote the common interests of environmental protection and economic development.

## 5. Conclusion

China is a big agricultural country, and the development of agriculture is beneficial to China's economic development. With the increasing international status of China, agricultural products are also popular in the liberalization of international trade, but the economic development also faces challenges. The agricultural environment has been seriously damaged, which has affected the development of agricultural products, which has led to the slow process of international agricultural trade liberalization. Therefore, a significant influence on the growth of agricultural trade liberalization is the study of the sustainable development of the agricultural environment and ensuring that it can achieve sustainable development. This research conducts a thorough assessment of the sustainable development of the agricultural environment using the emergy ecological footprint model and puts forward corresponding measures. After investigation and analysis in the experimental part, it is found that China's agricultural products have developed in international trade in recent years, indicating that the status of agricultural products in the world is also getting higher and higher. The experiment compares and analyzes the ecological footprint model and the emergy ecological footprint model and finds that the evaluation of the emergy ecological footprint model is more comprehensive and accurate. Finally, it is concluded that the development of international free trade of agricultural products will be more and more smooth only if the agricultural environment has been developed sustainably. The evaluation method proposed in this paper is within the scope of people's knowledge, and there may be better evaluation methods, which need to be studied in future work. It will also constantly correct its shortcomings.

## Figures and Tables

**Figure 1:** Agricultural sustainability.

**Figure 2:** Agricultural environment.

**Figure 3:** Agricultural Sustainability Index figure.

**Figure 4:** Ecological footprint analysis.

**Figure 5:** Income of major agricultural products and employment of farmers from 2014 to 2018.

**Figure 6:** Farmer employment from 2014 to 2018.

**Figure 7:** Effective utilization of fertilizers.

**Figure 8:** Agricultural environmental damage rate in province A.

**Table 1:** Import value of agricultural products (growth rate) from 2014 to 2018.

Year	Cereals	Vegetable	Fruit	Livestock products
2014	9.6%	11.9%	13.7%	16.2%
2015	11.8%	17.4%	17.6%	18.5%
2016	13.6%	15.9%	19.8%	19.4%
2017	18.9%	22.7%	26.5%	22.5%
2018	21.7%	25.6%	31.8%	23.3%

**Table 2:** 2014-2018 agricultural product export value (growth rate).

Year	Cereals	Vegetable	Fruit	Livestock products
2014	5.7%	8.7%	11.9%	15.5%
2015	10.6%	18.8%	18.6%	17.8%
2016	17.9%	19.4%	21.3%	23.2%
2017	25.4%	25.3%	26.8%	29.0%
2018	33.2%	35.5%	33.0%	30.8%

**Table 3:** Annual chemical fertilizer usage in the country and province A from 2014 to 2018.

Year	National fertilizer use (10,000 tons)	Fertilizer usage in province A (10,000 tons)	National average fertilizer usage (kg/ha)	Average fertilizer usage in province A (kg/ha)
2014	10879.4	3647.2	1643.4	4352.5
2015	12785.7	3748.9	1785.6	5636.3
2016	14638.5	3980.6	2175.8	6590.4
2017	16890.6	4325.3	2687.5	7825.1
2018	19536.2	4880.9	3636.2	8903.6
2019	23245.5	5256.4	4245.9	8094.5

## Data Availability

The datasets generated during and/or analyzed during the current study are not publicly available due to sensitivity and data use agreement.
